RETRACTED

# Genome-Wide Analysis of the Dof Transcription Factor Gene Family Reveals Soybean-Specific Duplicable and Functional Characteristics

**DOI:** 10.1371/journal.pone.0076809

**Published:** 2013-09-30

**Authors:** Yong Guo, Li-Juan Qiu

**Affiliations:** The National Key Facility for Crop Gene Resources and Genetic Improvement (NFCRI)/Institute of Crop Science, Chinese Academy of Agricultural Sciences, Beijing, P. R. China; Key Laboratory of Horticultural Plant Biology (MOE), China

## Abstract

The Dof domain protein family is a classic plant-specific zinc-finger transcription factor family involved in a variety of biological processes. There is great diversity in the number of *Dof* genes in different plants. However, there are only very limited reports on the characterization of Dof transcription factors in soybean (*Glycine max*). In the present study, 78 putative *Dof* genes were identified from the whole-genome sequence of soybean. The predicted *GmDof* genes were non-randomly distributed within and across 19 out of 20 chromosomes and 97.4% (38 pairs) were preferentially retained duplicate paralogous genes located in duplicated regions of the genome. Soybean-specific segmental duplications contributed significantly to the expansion of the soybean *Dof* gene family. These Dof proteins were phylogenetically clustered into nine distinct subgroups among which the gene structure and motif compositions were considerably conserved. Comparative phylogenetic analysis of these Dof proteins revealed four major groups, similar to those reported for *Arabidopsis* and rice. Most of the *GmDofs* showed specific expression patterns based on RNA-seq data analyses. The expression patterns of some duplicate genes were partially redundant while others showed functional diversity, suggesting the occurrence of sub-functionalization during subsequent evolution. Comprehensive expression profile analysis also provided insights into the soybean-specific functional divergence among members of the Dof gene family. *Cis*-regulatory element analysis of these *GmDof* genes suggested diverse functions associated with different processes. Taken together, our results provide useful information for the functional characterization of soybean *Dof* genes by combining phylogenetic analysis with global gene-expression profiling.

## Introduction

The transcriptional regulation of gene expression influences or controls many important cellular processes, such as signal transduction, morphogenesis, and environmental stress responses [1]. Transcription factors (TFs) are a group of proteins that control cellular processes by regulating the expression of downstream target genes [2]. Therefore, the identification and functional characterization of TFs is essential for the reconstruction of transcriptional regulatory networks [3]. In plants, ~60 families of TFs have been identified based on bioinformatics analysis and manual inspection [4,5]. The *Arabidopsis* genome codes for at least 1533 TFs, which account for about 5.9% of its estimated total number of genes [1]. As for soybean (*Glycine max*), ~12.2% of the 46,430 predicted protein-coding loci have been identified to encode 5,671 putative TFs [6].

RETRACTED

The Dof (DNA binding with one finger) TF family belongs to a class of plant-specific TFs that are not found in other eukaryotes such as yeast, *Caenorhabditis elegans*, *Drosophila* , fish or humans [7]. Bioinformatics analysis predicts 36 *Dof* genes in the *Arabidopsis* genome and 30 in the rice genome [8], while 41 have been described in poplar [9], 31 in wheat [10], and 28 in sorghum [11]. Dof protein is characterized by an N-terminal Dof domain of 50-52 amino-acid residues structured as a Cys2/Cys2 (C2/C2) zinc finger that recognizes a *cis*-regulatory element containing the common core sequence 5’-

(T/A)AAAG-3’ [12-14]. The Dof domain is bifunctional, mediating both DNA-protein and protein-protein interactions. Different Dof TFs may form homo- and/or hetero-dimeric complexes through the Dof domain in a given cell type and have various functions, acting as positive or negative regulators of their targets [15,16]. Other than the conserved Dof domain, diversified transcriptional regulation domains are also located at the C-terminal regions of Dof proteins. The conserved Dof domain might endow all Dof domain proteins with similar characteristics, while the diversified regions outside the Dof domain might be linked to the different functions of distinct Dof domain proteins [14].

Dof TFs are associated with many plant-specific physiological processes related to stress responses, photosynthesis, growth and development [17-27]. In *Arabidopsis* , some of the well-characterized *Dof* genes include *DAG1* and *DAG2* which are associated with seed germination [17,28], and *CDF1*, *CDF2* and *CDF3* which are involved in the photoperiodic control of flowering [19]. Some of the *Dof* TF genes (*AtDof2.4*, *AtDof5.8* and *AtDof5*.*6*/*HCA2*) are reported to be expressed specifically in cells at an early stage of vascular tissue development [18,29]. In rice, *OsDof3* is involved in gibberellins-regulated expression [30]. Maize *Dof1* and *Dof2* are activators of gene expression associated with carbohydrate metabolism, including the gene encoding phosphoenolpyruvate carboxylase [25,27]. In wheat, the Dof TF gene *WPBF* functions both during seed development and other growth and development processes [31]. A Dof gene, *StDof1*, which is expressed in epidermal fragments highly-enriched in guard cells, interacts in a sequence-specific manner with a *KST1* promoter fragment containing the TAAAG motif in tomato [12]. Some *Dof* TF genes also take part in the stress and defense responses of plants. Previous study showed that the RNA expression levels of three *Dof* genes (*OBP1*, *OBP2*, and *OBP3*) increase following treatment with auxin, salicylic acid or cycloheximide, while the OBP proteins have similar *in vitro* DNA-binding properties and are able to interact with OBF4, a bZIP transcription factor [32]. In response to drought treatment, some *TaDof* genes are down-regulated and two of them (*TaDof14* and *TaDof15*) are significantly upregulated, indicating that these genes may be involved in drought adaptation [10].

RETRACTED

Although quite a few Dof TFs have been functionally characterized in the model plant *Arabidopsis* and others, the functions of most members of the Dof family remain unknown. Especially in soybean, the typical legume species, there are only very limited reports on the functional characterization of Dof TFs. Wang et al. (2006) identified 28 GmDof proteins with recognizable Dof domain from 39 putative unigenes for the *Dof* gene family after analysis of their Expressed Sequence Tags (ESTs) in soybean [33,34] and detailed study of two *GmDof* genes suggested they increased the content of total fatty-acids and lipids in transgenic *Arabidopsis* by upregulating genes that were associated with fatty-acid biosynthesis [34]. Completion of the soybean genome greatly facilitated the identification of gene families at the whole-genome level [6]. In the present study, a genome-wide identification of Dof domain TFs in soybean was performed and revealed an expanded Dof family with 78 members.

Detailed analysis of the sequence phylogeny, genome organization, gene structure, conserved motifs, duplication status, expression profiling, and *cis*-elements was performed. It is noteworthy that nearly all of the *GmDof* genes (38 pairs) were preferentially-retained duplicates located in duplicated regions of the genome, indicating soybean-specific duplicable characteristics of the *Dof* gene family in this species. The putative soybean-specific functions of the predicted *GmDof* genes were investigated by analyzing the expression profiles using RNA-seq data and *cis*-regulatory elements associated with these genes in the promoter region. Our data provide a basis for the further evolutionary and functional characterization of the *Dof* gene family in soybean.

## Materials and Methods

### Database search and sequence retrieval

The Dof sequences of *Arabidopsis thaliana* and *Oryza sativa* were downloaded from the *Arabidopsis* genome TAIR release 9.0 (http://www.arabidopsis.org/) and the rice genome annotation database (http://rice.plantbiology.msu.edu/, release 5.0). The amino-acid sequence of the Dof domain was used to search for potential Dof-domain homolog hits in the whole-genome sequence of *G. max* with BLASTP at the Phytozome database (http:/www.phytozome.net) [35]. All non-redundant hits with expected values <1E-5 were collected and compared with the Dof family in PlantTFDB (http://planttfdb.cbi.edu.cn/) [5] and LegumeTFDB (http://legumetfdb.psc.riken.jp/) [36]. As for the incorrectly-predicted genes, manual re-annotation was performed using the on-line web server GENSCAN (http://genes.mit.edu/GENSCAN.html) [37] and/or RT-PCR cloning. The re-annotated sequences were further manually analyzed to confirm the presence of the Dof domain using the InterProScan program (http://www.ebi.ac.uk/Tools/InterProScan/) [38].

RETRACTED

### Protein Alignment and Phylogenetic Analysis

Multiple sequence alignments of the full-length deduced amino-acid sequences of Dof proteins were performed by Clustal X (version 1.83) [39]. The distribution of amino-acid residues at the corresponding positions in domain profiles for the conserved Dof domains of GmDofs were created using WebLogo [40]. Unrooted phylogenetic trees were constructed with MEGA 4.0 using the Neighbor-Joining (NJ) method and the bootstrap test carried out with 1000 iterations [41]. The pairwise gap deletion mode was used to ensure that the more divergent C-terminal domains could contribute to the topology of the NJ tree.

### Genomic structure and chromosomal location

The Gene Structure Display Server program [42] was used to illustrate the exon/intron organization for individual *Dof* genes by comparison of the coding sequences with their corresponding genomic DNA sequences from Phytozome (http://www.phytozome.net/gmax). The chromosomal locations of soybean *Dofs* were mapped to the duplicated blocks using the CViT (Chromosome Visualization Tool) genome search and synteny viewer at the Legume Information System (http://comparative-legumes.org/) [43,44]. The deduced amino-acid sequences of all *GmDofs* were used to search against the soybean genome and the results were displayed using CViT.

### Calculation of Ks and Ka to date duplication events

Clustal X (version 1.83) was used to make pairwise alignments of the paralogous nucleotide sequences [39]. Ks (synonymous substitution rate) and Ka (non-synonymous substitution rate) were estimated using the program DnaSp v5 [45]. The Ks values were then used to calculate the approximate date of duplication event (T = Ks/2λ), assuming a clock-like rate (λ) of synonymous substitution of 6.1×10^−9^ substitutions/synonymous site/year for soybean [6,46,47].

RETRACTED

### Identification of conserved motifs

The deduced amino-acid sequences of the 78 *GmDofs* were analyzed by MEME (Multiple EM for Motif Elicitation) version 4.9.0 (http://meme.nbcr.net/meme/cgi-bin/meme.cgi) [48] for motif analysis. To identify conserved motifs in these sequences, selection of the maximum number of motifs was set to 30 with a minimum width of 6 and a maximum width of 200 amino-acids, while other factors were set at default values. Structural motif annotation was performed using the SMART (http://smart.embl-heidelberg.de) [49] and Pfam (http://pfam.sanger.ac.uk) databases [50].

### Expression analysis of soybean Dof genes

The genome-wide transcriptome data from seeds during several stages of development and throughout the soybean life cycle (obtained with high-throughput sequencing) were downloaded from the NCBI database (http://www.ncbi.nlm.nih.gov; accession numbers SRX062325–SRX062334). The transcript data were obtained from seeds at five stages of development (globular, heart, cotyledon, early-maturation, and dry seeds), vegetative tissue (leaves, roots, stems, and whole seedlings), and reproductive tissue (floral buds). All transcript data were analyzed with Cluster 3.0 [51] and the heat map was viewed in Java Treeview [52].

### Cis-regulatory element analysis

For promoter analysis, 1000-bp sequences upstream from the initiation codon of the putative *GmDofs* were retrieved. These sequences were then subjected to search in the PLACE database (http://www.dna.affrc.go.jp/PLACE/signalscan.html) [53] to identify *cis*-regulatory elements.

## Results and Discussion

### Identification of Dof-encoding gene family in soybean

In order to identify the *Dof* gene family in the soybean genome, the amino-acid sequence of the conserved Dof domain was used to perform a BLAST search against the *Glycine max* v1.1 genome (http://www.phytozome.net). A total of 79 non-redundant *Dof* transcription factor-encoding genes were identified from the whole genome. The presence of the conserved Dof domain in the predicted GmDof protein was a typical feature for consideration as a member of the Dof TF family. To verify the reliability of our results, all of the putative Dof protein sequences were subjected to functional analysis by InterProScan. A typical zinc-finger Dof-type profile was found in all *GmDof*-encoding genes except for one, annotated as *Glyma08g12230*, which appears to be a pseudogene owing to a stop codon within the Dof domain.

The 78 soybean *Dof* genes were numbered from *GmDof01.1* to *GmDof20.2* following the nomenclature proposed for *Arabidopsis* and according to their positions on different chromosomes. The identified *GmDof* genes encode peptides ranging from 147 to 555 amino-acids in length with an average of 335. The detailed information of the Dof family genes in soybean, including accession numbers and similarities to their *Arabidopsis* orthologs, as well as nucleotide and protein sequences, are listed in Table 1 and Additional Table S1. The Dof gene family in soybean is largest compared with the estimates for other plant species, which range from ~36 in *Arabidopsis* [13], ~30 in rice [8], ~28 in sorghum [11] and ~27 in *Brachypodium* *distachyon* [54]. The member of *Dof* genes in soybean is roughly 2.4-fold that in *Arabidopsis* , which is consistent with the ratio of 1.4-1.6 putative *Populus* homologs for each *Arabidopsis* gene, based on comparative genomics studies [9]. This ratio is almost consistent with that among all the putative protein coding genes of these three species, although the genome size of soybean (1,115 Mb) is almost 9.7 times that of *Arabidopsis* (115 Mb) and 2.3 times that of *Populus* (480 Mb) [6,55,56].

RETRACTED

**Table 1:** Summary of Dof family members in soybean.

**Gene Symbol**	**Gene Locus**	**Gene Location**	**Amino Acids**	**Introns**	**Score**	**E-value**
*GmDof01.1*	*Glyma01g02610*	Gm01: 2137617-2139436	337	0	106.4	8.00E-24
*GmDof01.2*	*Glyma01g05960*	Gm01: 5750259-5754433	479	1	92.0	4.00E-20
*GmDof01.3*	*Glyma01g38970*	Gm01: 50951027-50952807	336	0	104.4	3.10E-23
*GmDof02.1*	*Glyma02g06970*	Gm02: 5595711-5596415	234	0	96.7	5.50E-21
*GmDof02.2*	*Glyma02g10250*	Gm02: 8123065-8125204	371	1	101.3	2.30E-22
*GmDof02.3*	*Glyma02g12081*	Gm02: 10302501-10306472	485	1	95.9	1.00E-20
*GmDof02.4*	*Glyma02g35296*	Gm02: 40034736-40035659	307	0	102.1	1.60E-22
*GmDof03.1*	*Glyma03g01030*	Gm03: 756237-758785	472	1	92.8	9.20E-20
*GmDof03.2*	*Glyma03g41980*	Gm03: 47319684-47321893	257	0	105.1	1.70E-23
*GmDof04.1*	*Glyma04g31690*	Gm04: 35880682-35882596	341	0	99.8	8.00E-22
*GmDof04.2*	*Glyma04g33410*	Gm04: 39029262-39032664	470	1	100.5	4.30E-22
*GmDof04.3*	*Glyma04g35650*	Gm04: 42048974-42051454	344	1	110.2	5.50E-25
*GmDof04.4*	*Glyma04g41170*	Gm04: 47030349-47032300	297	1	105.1	1.80E-23
*GmDof04.5*	*Glyma04g41830*	Gm04: 47667211-47668500	289	0	110.5	4.30E-25
*GmDof05.1*	*Glyma05g00970*	Gm05: 586599-589518	473	1	98.2	2.00E-21
*GmDof05.2*	*Glyma05g02220*	Gm05: 1636697-1639230	330	1	105.5	1.30E-23
*GmDof05.3*	*Glyma05g07460*	Gm05: 7516304-7518205	292	0	104.8	2.00E-23
*GmDof05.4*	*Glyma05g29090*	Gm05: 34760928-34763043	165	1	92.0	1.60E-19
*GmDof06.1*	*Glyma06g12950*	Gm06: 10094214-10095083	289	0	112.1	1.40E-25
*GmDof06.2*	*Glyma06g13671*	Gm06: 10805902-10807867	206	1	104.8	2.40E-23
*GmDof06.3*	*Glyma06g19330*	Gm06: 15557061-15559563	353	1	108.2	2.00E-24
*GmDof06.4*	*Glyma06g20950*	Gm06: 17335571-17338829	458	1	100.9	2.90E-22
*GmDof06.5*	*Glyma06g22797*	Gm06: 19579399-19580371	303	1	99.8	6.80E-22
*GmDof07.1*	*Glyma07g01461*	Gm07: 936400-938618	211	0	98.6	1.40E-21
*GmDof07.2*	*Glyma07g05950*	Gm07: 4649017-4651265	281	0	107.1	4.90E-24
*GmDof07.3*	*Glyma07g31340*	Gm07: 36361704-36363720	332	0	97.1	4.70E-21
*GmDof07.4*	*Glyma07g31860*	Gm07: 36820811-36821677	288	0	93.2	7.60E-20
*GmDof07.5*	*Glyma07g31870*	Gm07: 36829670-36831859	348	1	103.2	6.90E-23
*GmDof07.6*	*Glyma07g35690*	Gm07: 41004726-41008389	479	1	97.1	5.20E-21
*GmDof08.1*	*Glyma08g20840*	Gm08: 15829658-15831897	213	0	93.6	5.80E-20
*GmDof08.2*	*Glyma08g24591*	Gm08: 18749907-18753887	463	1	95.1	1.70E-20
*GmDof08.3*	*Glyma08g37530*	Gm08: 36252447-36254191	403	0	105.9	9.00E-24
*GmDof08.4*	*Glyma08g47290*	Gm08: 46169187-46171177	367	1	108.6	1.50E-24
*GmDof09.1*	*Glyma09g33350*	Gm09: 39841007-39842035	342	0	105.9	9.00E-24
*GmDof09.2*	*Glyma09g37170*	Gm09: 42705807-42709793	503	1	91.7	2.00E-19
*GmDof10.1*	*Glyma10g10142*	Gm10: 9742414-9743975	309	0	102.4	1.10E-22
*GmDof10.2*	*Glyma10g31700*	Gm10: 40190913-40205863	324	1	103.2	6.80E-23
*GmDof11.1*	*Glyma11g06300*	Gm11: 4474891-4476607	339	0	104.0	3.70E-23
*GmDof11.2*	*Glyma11g14920*	Gm11: 10654917-10656815	288	1	104.0	4.30E-23
*GmDof11.3*	*Glyma11g15761*	Gm11: 11423453-11425703	310	1	101.7	2.10E-22
*GmDof12.1*	*Glyma12g06880*	Gm12: 4679868-4681949	307	1	104.0	3.40E-23
*GmDof12.2*	*Glyma12g07710*	Gm12: 5322929-5325618	305	1	107.8	2.90E-24
*GmDof13.1*	*Glyma13g05480*	Gm13: 5801463-5804791	488	1	96.3	7.60E-21
*GmDof13.2*	*Glyma13g24600*	Gm13: 27964926-27967177	353	1	102.1	1.50E-22
*GmDof13.3*	*Glyma13g24611*	Gm13: 27973342-27974271	309	0	96.7	6.50E-21
*GmDof13.4*	*Glyma13g25120*	Gm13: 28389200-28391375	336	0	97.1	4.80E-21
*GmDof13.5*	*Glyma13g30331*	Gm13: 33007956-33010080	147	1	86.3	8.00E-18
*GmDof13.6*	*Glyma13g31100*	Gm13: 33571320-33573635	357	1	103.2	6.30E-23
*GmDof13.7*	*Glyma13g31110*	Gm13: 33583810-33584763	317	0	102.1	1.40E-22
*GmDof13.8*	*Glyma13g31560*	Gm13: 33969725-33970600	278	0	93.2	6.00E-20
*GmDof13.9*	*Glyma13g40420*	Gm13: 40913246-40915457	285	1	104.0	3.80E-23
*GmDof13.10*	*Glyma13g41031*	Gm13: 41429101-41431274	269	1	102.4	1.10E-22
*GmDof13.11*	*Glyma13g42820*	Gm13: 42682406-42684307	212	0	103.2	5.80E-23
*GmDof15.1*	*Glyma15g02620*	Gm15: 1777967-1779680	211	0	103.2	7.00E-23
*GmDof15.2*	*Glyma15g04430*	Gm15: 3099789-3101706	304	1	102.8	8.70E-23
*GmDof15.3*	*Glyma15g04980*	Gm15: 3568928-3571019	285	1	101.3	2.50E-22
*GmDof15.4*	*Glyma15g07730*	Gm15: 5453626-5455994	285	0	93.2	6.70E-20
*GmDof15.5*	*Glyma15g08230*	Gm15: 5800695-5803209	313	0	102.1	1.40E-22
*GmDof15.6*	*Glyma15g08250*	Gm15: 5817356-5819506	353	1	109.8	6.50E-25
*GmDof15.7*	*Glyma15g08860*	Gm15: 6264258-6266252	153	1	86.3	8.00E-18
*GmDof15.8*	*Glyma15g29870*	Gm15: 32718091-32721358	464	1	93.2	7.10E-20
*GmDof16.1*	*Glyma16g02550*	Gm16: 2119565-2121907	276	0	107.1	4.90E-24
*GmDof16.2*	*Glyma16g26030*	Gm16: 30193624-30194977	236	0	94.7	2.00E-20
*GmDof17.1*	*Glyma17g08950*	Gm17: 6612406-6614430	300	0	99.4	9.30E-22
*GmDof17.2*	*Glyma17g09710*	Gm17: 7203819-7206839	330	1	108.6	1.70E-24
*GmDof17.3*	*Glyma17g10920*	Gm17: 8207249-8210723	471	1	99.4	0.0
*GmDof17.4*	*Glyma17g21540*	Gm17: 20917544-20919496	352	0	105.5	1.30E-23
*GmDof18.1*	*Glyma18g26870*	Gm18: 30922106-30923215	369	0	104.4	2.90E-23
*GmDof18.2*	*Glyma18g38560*	Gm18: 46153747-46155733	363	1	102.8	9.20E-23
*GmDof18.3*	*Glyma18g49520*	Gm18: 58916821-58920915	501	1	95.1	1.70E-20
*GmDof18.4*	*Glyma18g52661*	Gm18: 61211505-61213733	363	1	102.4	1.20E-22
*GmDof19.1*	*Glyma19g02710*	Gm19: 2647356-2650816	385	1	97.1	4.90E-21
*GmDof19.2*	*Glyma19g29610*	Gm19: 37285687-37288840	483	1	90.9	3.00E-19
*GmDof19.3*	*Glyma19g38660*	Gm19: 45513027-45514071	271	0	104.0	4.00E-23
*GmDof19.4*	*Glyma19g38750*	Gm19: 45606704-45607516	270	0	99.4	8.40E-22
*GmDof19.5*	*Glyma19g44670*	Gm19: 50031772-50033750	252	0	102.8	7.40E-23
*GmDof20.1*	*Glyma20g04600*	Gm20: 4815565-4819043	482	1	95.5	1.20E-20
*GmDof20.2*	*Glyma20g35910*	Gm20: 44105729-44107846	300	1	103.2	5.70E-23

To investigate the features of the homologous domain sequences, and the frequency of the most prevalent amino-acids at each position within the soybean Dof domain, multiple-alignment analysis using the amino-acid sequences of the Dof domains from 78 GmDofs was performed. In general, the basic regions of the Dof domains had 52 basic residues. The distribution of amino-acid residues at the corresponding positions of the soybean Dof domains also revealed that it was very similar to that of *Arabidopsis* , as expected from the evolutionary distances among plants (Figure 1). The Dof domain of soybean revealed highly-conserved sequences and 26 out of 52 amino-acids were 100% conserved in all GmDof proteins, including four absolutely-conserved cysteine residues that presumably coordinate zinc ion. Other highly conserved residues in the soybean Dof domains were Pro-4, Arg-5, Ser-8, Thr-11, Lys-12, Phe-13, Cys-14, Tyr-15, Asn-17, Asn-18, Tyr-19, Gln-23, Pro-24, Arg-25, Arg-33, Trp-35, Thr-36, Gly-38, Gly-39, Arg-42, Gly-47 and Gly-49. These highly-conserved residues were also nearly identical to the Dof domain proteins of other plants such as sorghum and tomato [11,57]. Moreover, five other amino-acid residues showed variation in less than three sequences among all *GmDofs*.

RETRACTED

**Figure 1:** Dof domains are highly conserved across all Dof proteins in soybean. The sequence logos are based on alignments of all soybean Dof domains. Multiple alignment analysis of 78 typical soybean Dof domains was performed with ClustalW. The bit score indicates the information content for each position in the sequence. Asterisks indicate the conserved cysteine residues (Cys) in the Dof domain.

### Phylogenetic Relationships and Gene Structure of Soybean Dof Genes

To examine the phylogenetic relationships among the Dof domain proteins in soybean, an unrooted tree was constructed from alignments of the full-length amino-acid sequences of all GmDof proteins (Figure 2A). The observed sequence similarity and phylogenetic tree topology allowed us to classify the soybean Dof gene family into nine subgroups (subgroups I-IX). Each subgroup had 4-19 members and the very high bootstrap value in each subgroup suggested a common origin for the *Dof* genes in each subgroup. Inspection of the phylogenetic tree topology revealed several pairs of Dof proteins with a high degree of homology in the terminal nodes of each subgroup, suggesting that they are putative paralogous pairs (Figure 2A). A total of 38 pairs of putative paralogous Dof proteins were identified, accounting for nearly the entire family (except for GmDof17.4 and GmDof05.4), with sequence identity ranging from 72% to 97% (see Additional Table S2 for details). So many putative paralogous Dof proteins supported the hypothesis that they evolved from a recent soybean genome duplication event [58].

**Figure 2:** Phylogenetic relationships and gene structure of soybean *Dof* genes. (A) The phylogenetic tree of soybean Dof proteins constructed from a complete alignment of 78 GmDof proteins using MEGA 4.0 by the neighbor-joining method with 1,000 bootstrap replicates. Percentage bootstrap scores >50% are indicated on the nodes. The nine major phylogenetic subgroups designated I to IX are indicated. (B) Exon/intron structures of *Dof* genes from soybean. Exons are represented by green boxes and introns by black lines. The sizes of exons and introns can be estimated using the scale below.

It is well known that gene structural diversity is a possible mechanism for the evolution of multigene families. In order to gain further insight into the structural diversity of Dof genes, we compared the exon/intron organization in the coding sequences of individual Dof genes in soybean. A detailed illustration of the exon/intron structures is shown in Figure 2B. According to their predicted structures, 35 of the *GmDof* genes have no introns whereas 38 contain one intron generally placed up-stream of the Dof domain, except for five (*GmDof10.2*, *GmDof20.2*, *GmDof13.5*, *GmDof15.7*, and *GmDof05.4*) with a down-stream intron. These exon/intron structures are similar to those of *Arabidopsis* , rice, and other plants [8,11,54]. The most closely-related members in the same subgroup generally showed the same exon/intron pattern, with the position and length of the intron almost completely conserved within most subgroups (Figure 2). For instance, the *Dof* genes in subgroups II, IV, VII and VIII all lacked an intron, while all members of subgroups III and IX contained one intron. In contrast, the gene structure appeared to be more variable in subgroups I, V and VI, which had the largest numbers of exon/intron structural variants with striking distinctions.

RETRACTED

### Chromosomal location and duplication of soybean Dof genes

Genome chromosomal location analyses revealed that *GmDofs* were non-randomly distributed on 19 of the 20 chromosomes (Figure 3). Nearly all *GmDof* genes were distributed on the chromosome arms while none were on the heterochromatin regions around the centromeric repeats. Among these chromosomes, chromosome 13 contained the largest number of eleven *Dof* genes followed by eight on chromosome 15. In contrast, no *Dof* genes were found on chromosome 14 and only two occurred on six chromosomes (chromosome 03, 09, 10, 12, 16, and 20). Substantial clustering of *Dof* genes was evident on several chromosomes, especially on those with high densities of the genes. For example, *GmDof07.4* and *GmDof07.5* located in an 8.8-kb segment on chromosome 07, while *GmDof15.5* and *GmDof15.6* located within a 19-kb segment on chromosome 15. Similarly, four genes (*GmDof13.2* and *13.3*, and *GmDof13.6* and *13.7*) were arranged in two clusters in 10-kb and 13-kb segments on chromosome 13 respectively (Figure 3).

**Figure 3:** Chromosomal locations, region duplications, and predicted clusters for soybean *Dof* genes. The schematic diagram of genome-wide chromosome organization and segmental duplication arising from the genome duplication event in soybean was derived from the CViT genome search and synteny viewer at the Legume Information System (http://comparative-legumes.org). Colored blocks to the left of each chromosome show duplications with chromosomes of the same color. For example, the gray blocks at the bottom of Gm10 correspond with regions on the brown Gm20, and *vice* *versa*. The chromosomal positions of all *Dof* genes in soybean were mapped on each chromosome. The locations of centromeric repeats are shown as black rectangles over the chromosomes. The chromosome numbers are indicated at the top of each bar and sizes of chromosomes are represented by the vertical scale.

RETRACTED

Segmental duplication, tandem duplication, and transposition events are the main causes of gene-family expansion. Two or more genes located on the same chromosome confirms a tandem duplication event, while gene duplication on different chromosomes is designated a segmental duplication event [59]. Previous studies revealed that the soybean genome has undergone at least two rounds of genome-wide duplication followed by multiple segmental duplication, tandem duplication, and transposition events such as retroposition and replicative transposition [58]. To detect a potential relationship between putative paralogous pairs of soybean *Dofs* and potential segmental duplications, the *Dof* genes were mapped to the duplicated blocks using the CViT genome search and synteny viewer at the Legume Information System (http://comparative-legumes.org/) [43,44]. The distributions of *Dof* genes relative to the corresponding duplicate genomic blocks are illustrated in Figure 3. Within the duplicated blocks associated with a duplication event, 22 out of 38 putative paralogous pairs were preferentially-retained duplicates that were located in a segmental duplication of a long fragment (>1 Mb), and 13 putative paralogous pairs were located in a segmental duplication of a short fragment (<1 Mb) (Table 2). Another two putative paralogous pairs lacked the corresponding duplicates and only one putative paralogous pair (*GmDof19.3/19.4*) was possibly due to tandem duplication in the same orientation. These results implied that segmental duplication was predominant for *Dof* gene evolution in soybean, and that tandem duplication was involved. This relationship between soybean *Dofs* and potential segmental duplications suggests that dynamic changes occurred following segmental duplication, leading to loss of some of the genes.

**Table 2:** Duplicated *Dof* genes in soybean and the dates of the duplication blocks.

**Gene 1**	**Gene 2**	**Fragment Duplication**	**Ka**	**Ks**	**Ka/Ks**	**Date (Mya)**
*GmDof07.3*	*GmDof13.4*	Small	0.0313	0.1010	0.3099	8.28
*GmDof07.5*	*GmDof13.2*	Small	0.0662	0.1355	0.4886	11.11
*GmDof13.6*	*GmDof15.6*	Large	0.0556	0.0951	0.5846	7.80
*GmDof07.4*	*GmDof13.3*	Small	0.0916	0.1079	0.8489	8.84
*GmDof13.7*	*GmDof15.5*	Large	0.0441	0.1205	0.3660	9.88
*GmDof02.2*	*GmDof18.4*	Small	0.0498	0.0938	0.5309	7.69
*GmDof13.10*	*GmDof15.2*	Large	0.0555	0.1133	0.4898	9.29
*GmDof08.3*	*GmDof18.1*	None	0.1244	0.3315	0.3753	27.17
*GmDof13.11*	*GmDof15.1*	Large	0.0424	0.1295	0.3274	10.61
*GmDof10.2*	*GmDof20.2*	Large	0.0615	0.1561	0.3940	12.80
*GmDof04.4*	*GmDof06.2*	Large	0.0496	0.1395	0.3556	11.43
*GmDof11.3*	*GmDof12.2*	Small	0.0369	0.1188	0.3106	9.74
*GmDof13.9*	*GmDof15.3*	Large	0.0379	0.1148	0.3301	9.41
*GmDof05.2*	*GmDof17.2*	Large	0.0406	0.1156	0.3512	9.48
*GmDof04.1*	*GmDof06.5*	None	0.0811	0.2524	0.3213	20.69
*GmDof04.5*	*GmDof06.1*	Large	0.0807	0.2125	0.3798	17.42
*GmDof02.4*	*GmDof10.1*	Small	0.0410	0.1334	0.3073	10.93
*GmDof03.1*	*GmDof19.2*	Small	0.0503	0.1633	0.3080	13.39
*GmDof08.2*	*GmDof15.8*	Small	0.0901	0.1474	0.6113	12.08
*GmDof07.6*	*GmDof20.1*	Small	0.0458	0.1444	0.3172	11.84
*GmDof05.1*	*GmDof17.3*	Large	0.0448	0.0732	0.6120	6.00
*GmDof13.1*	*GmDof19.1*	Large	0.0633	0.1013	0.6249	8.30

In order to trace the dates of the duplication blocks, the DnaSP program was used to estimate the Ks and Ka distances, as well as the Ka/Ks ratios. The approximate dates of duplication events were calculated using Ks. Table 2 shows the results of analysis of segmental and tandem duplication blocks. The segmental duplications of the *Dof* genes in soybean originated from 6.0 Mya (million years ago, Ks = 0.0732) to 27.17 Mya (Ks = 0.2018), with the mean of 11.90 Mya (Ks = 0.1452); the Ks of tandem duplication of *GmDof19.3* and *GmDof19.4* was 0.0111, dating the duplication event at 0.91 Mya. Since the soybean genome underwent two polyploidy events at 13 and 58 Mya, all the segmental duplications of the *GmDof* genes occurred around 13 Mya when *Glycine* -specific duplication occurred in the soybean genome. The Ka/Ks ratios of 15 segmental duplication pairs and one tandem duplication pair were <0.3, while the ratios of the other 22 segmental duplication pairs were all >0.3, suggesting that significant functional divergence of some *GmDof* genes might have occurred after the duplication events.

RETRACTED

### Phylogenetic analysis of the Dof gene family in soybean, *Arabidopsis* , and rice

To investigate the molecular evolution and phylogenetic relationships among the Dof domain proteins in soybean, *Arabidopsis* , and rice, the 78 predicted GmDof proteins were subjected to multiple sequence alignment along with 36 *Arabidopsis* and 30 rice Dof proteins, and an unrooted phylogenetic tree was constructed using the NJ method, based on the alignment of all the Dof amino-acid sequences (Figure 4, Additional Table S3). The NJ tree showed that all the Dof family proteins from the three higher plants were divided into four Major Clusters of Orthologous Groups (MCOG A, B, C, and D) and nine well-supported clades (Figure 4), similar to previous reports [8,13]. Among these, group C constituted the largest clade, containing 47 members and accounting for 32.6% of the total *Dof* genes, and the other three groups contained 25 (Group A), 30 (Group B), and 42 (Group D) members, respectively. In general, the Dof members demonstrated an interspersed distribution in most subfamilies, indicating that the expansion of *Dof* genes occurred before the divergence of soybean, *Arabidopsis* , and rice. Based on the phylogenetic tree, several putative orthologs (*GmDof06.3/AtDof5.6*, *OsDof-2/GmDof07.6* (*GmDof09.2*), *AtDof1.6/OsDof-10*, or *AtDof2.4/OsDof-16/GmDof13.10* (*GmDof15.2*)) and paralogs (*AtDof5.7/AtDof4.7*, *OsDof-13/OsDof-30*, *GmDof03.1/GmDof19.2*) were also identified.

**Figure 4:** Phylogenetic tree of all Dof domain containing proteins from soybean, *Arabidopsis* , and rice. The deduced full-length amino-acid sequences of 78 soybean, 36 *Arabidopsis* and 30 rice *Dof* genes were aligned by Clustal X 1.83 and the phylogenetic tree was constructed using MEGA 4.0 by the neighbor-joining method with 1,000 bootstrap replicates. Each Dof subgroup is indicated by a specific color.

Moreover, since most of the *Arabidopsis* Dof genes with similar functions showed a tendency to fall into one subgroup, soybean *Dof* genes in the same subgroup may have similar functions. In subgroup A, eight soybean *Dof* genes clustered with the *Arabidopsis* Dof genes *AtDof2.4*, *AtDof4.7*, *AtDof5.7* and *AtDof3.6*(*OBP3*) in subgroup B1, and these have been identified to be involved in tissue differentiation (vascular development, floral organ abscission, leaf blade polarity and growth regulation) [20,29,32,60,61]. About 19 GmDofs showed maximum similarity with AtDof5.5(CDF1), AtDof5.2(CDF2), AtDof3.3(CDF3), AtDof2.3(CDF4), AtDof1.10(CDF5), and AtDof1.5(COG1) of *Arabidopsis* representing subgroup D1, which are basically CDF (Cycling Dof Factor) proteins associated with the regulation of photoperiodic flowering time by repressing the *CONSTANS* gene [19,62]. Specifically, the *Arabidopsis* Dof proteins AtDof4.2, 4.3, 4.4 and 4.5 constitute the distinct subgroup C3 and OsDof-13, 24, 25, 30 constitute the distinct subgroup D3, similar to what has been reported in *Arabidopsis* and rice clusters C3 and D3 [8]. These sets of *Dof* genes might be exclusively present in *Arabidopsis*/rice as no apparent counterpart in soybean as well as other plants.

### Conserved motifs outside the Dof domain

To reveal the diversification of *Dof* genes in soybean, putative motifs were predicted by the program MEME (Multiple Em for Motif Elicitation), and a total of 30 conserved motifs were found in all the 78 Dof proteins (Figure 5). Motif 1 was uniformly present in all the Dof proteins and represents the conserved Dof domain. Moreover, a number of common motifs were found in all soybean Dofs (the amino-acid consensus sequence of each motif is listed in Additional Table S4). As expected, most of the closely-related members in the phylogenetic tree had common motif compositions. For example, there were no conserved motifs outside the Dof domain in Subgroup I, while motifs 2, 3, 4, 5, 6, 7, 9, 10, 12, 17, and 22 appeared in nearly all the members of subgroup IX. In other subgroups, motifs 8 and 15 were specific to subgroup III, motifs 20 and 24 were specific to subgroup IV, motifs 18 and 29 were specific to subgroup V, motifs 11, 21, 19, 23, and 30 were specific to subgroup VI, motif 13 was specific to subgroup VII, and motifs 25, 26 and 27 were specific to subgroup VIII. These similarities in motif patterns might be related to similar functions of the Dof proteins within the same subgroup.

RETRACTED

**Figure 5:** Schematic distributions of the conserved motifs among defined gene clusters. Motifs were identified by means of MEME software using the deduced amino-acid sequences of the 78 GmDofs. The relative position of each identified motif in all Dof proteins is shown. Multilevel consensus sequences for the MEME defined motifs are listed in Table S4.

### Expression pattern of Dof genes in soybean

Since high-throughput sequencing and gene expression analyses have been performed on many soybean tissues at various developmental stages, publicly-available RNA-Seq data is thought to be a useful resources for studying gene expression profiles. Distinct transcript abundance patterns were readily identifiable in the RNA-Seq dataset at NCBI. Nearly all *Dof* genes (except for three: *GmDof02.4*, *GmDof13.1*, and *GmDof19.3*) have sequence reads in at least one tissue, their universal expression also indicating the importance of Dof TFs. The expression profiles of the 75 *Dof* genes were analyzed as shown in Figure 6. Most of the *Dof* genes showed distinct tissue-specific expression patterns across the ten tissues examined. All of the *GmDofs* having expression profiles were clustered into nine groups based on their expression patterns. The genes in clusters A-I were mainly expressed in root/floral bud, root, root/globular embryo, floral bud/globular embryo, leaf/floral bud, floral bud, cotyledon/early-maturation embryo, heart/cotyledon embryo, and dry seed.

**Figure 6:** Heatmap of expression profiles for soybean *Dof* genes across different tissues. The genome-wide transcriptome data of soybean were generated from the NCBI database (accession numbers SRX062325–SRX062334). The expression data were gene-wise normalized and hierarchically clustered. The relative expression level of a particular gene in each row was normalized against the mean value. The color scale below represents expression values, green indicating low levels and red indicating high levels of transcript abundance. The sources of the samples were as follows: SDLG (whole seedlings 6 days after imbibition), LEAF (leaves), ROOT (roots), STEM (stems), FBUD (floral buds), GLOB (globular-stage embryos), HRT (heart-stage embryos), COT (cotyledon-stage embryos), EM (early maturation stage embryos), and DRY (dry soybean seeds).

RETRACTED

Detailed analysis of the expression patterns of *GmDofs* showed that some of the genes clustered in the same subgroup of the phylogenetic tree (Figure 2) had similar expression patterns, also indicating the existence of redundancy among the *Dof* genes in these subgroups. For example, all of the *GmDofs* in subgroup VII were mainly expressed in floral buds while all of genes in subgroup V were mainly expressed in root and/or globular embryo. Most of the genes in subgroup IX had dominant expression patterns in floral buds and/or globular embryo. However, some Dof members in the same subgroups also had totally different expression patterns, even among paralogous genes with high identity of amino-acid sequences. In subgroup I of the phylogenetic tree (Figure 2), there were five kinds of expression patterns among all eight GmDof members. Three of four pairs of paralogous genes (*GmDof07.3/13.4*, *GmDof07.5/13.2*, and *GmDof13.6/15.6*) had different expression patterns and one pair (*GmDof13.8/15.4*) was mainly expressed in floral buds and globular embryo. The genes in the same subgroup with different expression pattern, especially paralogous genes, also revealed their functional diversity despite these *Dof* genes had highly similar amino-acid sequences.

### *Cis*-regulatory element analysis

The transcription rate of a gene is determined by trans-acting TFs that bind to *cis*-regulatory elements in promoters, additional co-factors, and chromatin accessibility [63]. A common approach to identify functional *cis*-acting promoter elements is to discover over-represented motifs in co-expressed genes. It is assumed that promoter motifs conserved in clusters of co-expressed and functionally-related genes may be involved in mediating coordinated gene activity [64,65]. The promoter regions of the *GmDof* genes (1000-bp sequences upstream from the translational start site) were analyzed using the PLACE database to identify putative *cis*-elements. According to the PLACE results, many similar *cis*-acting regulatory DNA elements associated with root, leaf, flower, seed, nodulin, abiotic or biotic stress, and hormone (Additional Table S5) occurred in the promoter regions of the 78 *GmDof* genes. For example, *cis*-elements related to root-specific (ROOTMOTIFTAPOX1), leaf-specific (CACTFTPPCA1), and flower-specific (POLLEN1LELAT52) were present in all soybean *GmDof* promoters (Additional Table S5). Especially, all of the *GmDof* promoters contained Dof elements (DOFCOREZM) ranging from 4 to 37 copies, indicating the important role of Dof TFs in regulating themselves. Furthermore, the differences in common *cis*-elements across these promoter regions, including both number and distance from the start codon (Additional Table S5), indicated that the number of *cis*-elements and their distance from the start site affect the responsiveness of *GmDofs* to the environment and development.

RETRACTED

## Conclusions

Transcriptional regulation is an important mechanism underlying gene expression. The number, position and interaction between different *cis*-elements and the TFs at a given gene promoter determine the gene expression pattern. These TFs can be classified into gene families according to the presence of a particular DNA-binding domain. In this study, a comprehensive analysis was conducted and a multitude of *Dof* gene family members were identified in the soybean genome. Genome-wide analysis revealed the existence of 78 full-length *Dof* genes, and multiple sequence alignment of the GmDof proteins showed strong conservation of four cysteine residues and the other amino-acid residues in the Dof domains. Phylogenetic analysis revealed that all GmDofs were clustered into nine distinct subgroups. The exon/intron structure and motif composition of the *Dofs* were highly conserved in each subfamily, indicating their functional conservation. The *Dof* genes were non-randomly distributed within and across 19 chromosomes, and a high proportion of *GmDofs* were preferentially-retained duplicates located on duplicated blocks. Soybean-specific segmental duplications of the genome contributed significantly to the expansion of the soybean *Dof* gene family. The comparative phylogenetic analysis of soybean Dof proteins with *Arabidopsis* and rice Dof proteins revealed four Major Clusters of Orthologous Groups and nine well-supported clades. The global expression profile analysis provided insight into the soybean-specific functional divergence among members of the *Dof* gene family. A majority of *GmDofs* showed specific temporal and spatial expression patterns, based on RNA-seq data analyses. The expression patterns of duplicate genes were partially redundant or divergent. The *cis*-regulatory element analysis of the predicted *Dof* genes revealed differences in common *cis*-elements across these promoter regions including both their number and distance from the start codon. The results presented here provide information useful for the functional characterization of soybean gene families by combining phylogenetic analysis with global gene expression profiling.

RETRACTED

## Supporting Information

Table S1 **Complete list of soybean *Dof* gene sequences identified in the present study.** The list comprises 78 *GmDof* gene sequences. The amino-acid sequences were deduced from their corresponding coding sequences; the genomic DNA sequences were obtained from Phytozome. Most of the transcripts were based on the *Glycine* *max* v1.1 annotation and some were from v1.0. Some of the Dof genes were re-annotated based on GENESCAN, paralogous genes, and/or RT-PCR.
(XLS)

Table S2 **Pairwise identities between homologous pairs of *Dof* genes from soybean.** Pairwise identities and sequence alignments of the 38 homologous pairs identified from the soybean Dof family.
(XLS)

Table S3 **List of *Dof* genes from *A. thaliana* and *O. sativa* used for phylogenetic analysis.** The *Dof* sequences of *A. thaliana* and *O. sativa* were downloaded from *Arabidopsis* genome TAIR release 9.0 (http://www.Arabidopsis.org/) and those of *O. sativa* from the rice genome annotation database (http://rice.plantbiology.msu.edu/, release 5.0). The nomenclature is according to previous reports [8,13].
(XLS)

Table S4 **Multilevel consensus sequences for the MEME-defined motifs found among different Dof proteins from soybean.** Consensus amino-acid sequences obtained from analysis of the 78 soybean Dof proteins with MEME software. The motif numbers are equivalent to those described in Figure 5. Motif 1 corresponds to the Dof DNA-binding domain.
(XLS)

Table S5 **The *cis*-acting regulatory DNA elements of 78 GmDof promoters.** The motifs of the soybean *GmDof* promoters were predicted by PLACE (http://www.dna.affrc.go.jp/PLACE/). The numbers show the occurrence frequency of the motifs in one promoter. The sequences were from the 1-kb sequence upstream of the ATG.
(XLS)
